# Stress Classification by Multimodal Physiological Signals Using Variational Mode Decomposition and Machine Learning

**DOI:** 10.1155/2021/2146369

**Published:** 2021-08-26

**Authors:** Nilima Salankar, Deepika Koundal, Saeed Mian Qaisar

**Affiliations:** ^1^Department of Virtualization, School of Computer Science, University of Petroleum & Energy Studies (UPES), Dehradun, India; ^2^Electrical and Computer Engineering Department, Effat University, Jeddah 22332, Saudi Arabia; ^3^Communication and Signal Processing Lab, Energy and Technology Research Centre, Effat University, Jeddah 22332, Saudi Arabia

## Abstract

In this pandemic situation, importance and awareness about mental health are getting more attention. Stress recognition from multimodal sensor based physiological signals such as electroencephalogram (EEG) and electrocardiography (ECG) signals is a very cost-effective way due to its noninvasive nature. A dataset, recorded during the mental arithmetic task, consisting of EEG + ECG signals of 36 participants is used. It contains two categories of performance, namely, “Good” (nonstressed) and “Bad” (stressed) (Gupta et al. 2018 and Eraldeír et al. 2018). This paper presents an effective approach for the recognition of stress marker at frontal, temporal, central, and occipital lobes. It processes the multimodality physiological signals. The variational mode decomposition (VMD) strategy is used for data preprocessing and for the decomposition of signals into various oscillatory mode functions. Poincare plots (PP) are derived from the first eight variational modes and features from these plots have been extracted such as mean, area, and central tendency measure of the elliptical region. The statistical significance of the extracted features with *p* < 0.5 has been performed using the Wilcoxson test. The multilayer perceptron (MPLN) and Support Vector Machine (SVM) algorithms are used for the classification of stress and nonstress categories. MLPN has achieved the maximum accuracies of 100% for frontal and temporal lobes. The suggested method can be incorporated in noninvasive EEG signal processing based automated stress identification systems.

## 1. Introduction

Short-term mental fatigue results in reduced efficiency in workspace, whereas long-term mental fatigue may result into brain damage. Therefore, timely awareness about reasonable rate of mental fatigue is very crucial. Stress management is very necessary for successful and happy leading life. The population who can easily manage stress does exhibit their behavior in brain as well and can be easily captured by noninvasive approach. Acquisition of data in real time environment is very tough; thus, induced technique plays a very important role in behavioral study. Three levels of mental arithmetic tasks that are mostly used in literature are easy, medium, and hard and it is an appropriate technique for inducing the stress in virtual environment [1]. Nowadays, in every work domain and culture, performance setting is marked and stress management is a key to succeed and nonmanagement of stress not only leads to failure but is a major reason of depression, frustration, and negative approach towards life. Thus, stress management is an important skill to learn and to help this fraternity by early identification of markers which is very essential.

In literature, lot of attempts have been made in this direction. Firstly, in order to understand the markers of fraternity stress and nonstress, various types of studies have been conducted where arithmetic test is the most common technique which has been widely adopted. However, mental arithmetic task is an appropriate stress inducing technique but it has certain limitation and according to age it has shown different impact [2]. To capture the response from different types of subjects in response to various stress induced techniques, multimodality approach has exhibited significant role and its impact is noteworthy [3]. Various types of studies have been carried out in this domain and quite interesting study has been carried out on the arithmetic task where experimentation has been done on numbers with respect to ordered and unordered [4]. As brain has various lobes and it gives response to various activities, sometimes, it might be subject dependent and independent and this correlation has been identified by studying different regions of brain while performing activity abacus [5] and hemisphere activation has been studied [6]. Thinking also acts as a vital role in the generation of brain signals; thus, silent text reading and study of brain signals in response to silent text reading have been carried out [7–9].

For capturing the physiological signals in response to induced techniques, electroencephalogram (EEG), electromyography (EMG), electrooculography (EOG), and electrocardiography (ECG) have mostly been used whereas photoplethysmography (PPG) also serves a very important role in capturing physiological signals [3, 10]. Single channel study though focuses on single task whereas multimodal ones focus and capture the responses from various parts; thus, multimodality signals and their correlation with mental workload have been studied [11, 12]. Every significant activity contains the significance of various brain regions and its association details are presented [13]. Even though behavioral impact is available all over, certain lobes have shown prominent changes; majorly frontal region exhibits prominent changes in signals while performing mental arithmetic task [14]. Data acquisition by inducing relevant technique/protocol and its systematic analysis lead to designing of an appropriate study protocol and popularly used methods are appropriate selection of channels [15]. Analysis of an EEG signal from only visualization is an empirical science and needs expertise in neurological domain and thus, it is very time-consuming and tedious process [16]. As there are stress induced techniques, similarly stress relieving techniques and their cognitive impact are also great to understand [17]. Stress has significant impact to invoke and subsidize emotions [18] and generate different behavioral response in epilepsy patients [19, 20]. Physiological signals also help to learn behavioral pattern in special category [21]. In order to better visualize signals decomposition method, feature extraction plays very crucial role. Decomposition of signals in empirical way has been widely used [22], but high frequency study is well supported by VMD; thus authors have proposed the use of VMD technique to better visualize the signal in time domain while retaining its frequency components. This method has proven its significant role in area of seizure [23, 24]. Understanding of connectivity among brain regions gives clear insight about origin and exit of electrical connectivity between regions [20]. However, convolution techniques have been used [21] for reading EEG signals but they have no flexibility of reading signals in time-frequency domain and sometimes because of nonstationary behavior of the EEG signal they need to compromise on accuracy [25]. There are unlimited areas where stress gets evoked and reason for it could be noise trigger or unpleasant vision [26]. As it is said every task is time bounded and it is proven in studying correlation of activity and time in [24]. Mere clean data acquisition does not solve the purpose unless relevant features have been extracted and its importance is viable [1, 23]. Capturing of signal from throughout brain region is very tedious; thus, study of only frontal region has been carried out in [27]. EEG signals are very effective in carrying correlation between various rhythmic signals [28]. Activation of specific region and band is dependent upon types of activities performed by subjects [29, 30]. Because of scarcity of professional automation and semiautomation, the analysis of multimodal signals such as EEG + ECG is very important [31]. In real life, time requirement to induce stress and analyze its resistant capability has various constraints [32–34].

The main objective of this work is to extract relevant features from the multimodality physiological signals and to design a classifier which can easily detect the stress (bad) and nonstress (good) performer where signals have been captured while subjects have performed silent math activity as well as during getting acquainted with an environment. Therefore, key contributions of this research work are as follows:

(i) Proposing an effective method for the automated classification of stress resistant capability while conducting short time mental arithmetic task.
  1. The VMD is used for decomposing the multimodal physiological signals.
  2. The PPs plots are derived from the first eight variational modes.
  3. The discriminating features have been identified such as area, mean, and central tendency measure from each PP.
  4. The extracted features are passed to the considered classifiers for automated identification of good and bad classes.

Remainder of the paper is organized as follows: Section 2 describes materials and methods, Section 3 discusses the results, and conclusion is presented in Section 4.

## 2. Materials and Methods

This section has contributed for the discussion of methodology which consists of four components: (i) description of dataset used for an experimentation, (ii) selection of channels for an experiment purpose, (iii) VMD, (iv) PPs and features extraction, (v) classifiers, and (vi) evaluation measures.

The suggested work flow is shown in Figure 1. Different stages are described in the following subsections.

### 2.1. Dataset

In this work, dataset used for the purpose of an experimentation and evaluation of stress classifier is available publicly [15]. For each subject, two trails have been conducted where physiological signals (EEG + ECG) have been captured. Trail 1 is baseline activity for 180 seconds to get subjects acquainted with an environment and 60 seconds' data for actual cognitive task performance. Sampling rate for data acquisition is 516 Hz. Thus, each subject cognitive task has raw file with data dimension (21 channels x 516 samples x time duration results) into (21 × 516 × 60 = 650160) data points and (21 × 516 × 180 = 1950480) data points for baseline activity. Independent component analysis (ICA) has been done for the purpose of noise removal. However, dataset is captured while subjects were performing silent math activity where no muscle movement was expected but noise generally get introduced and elimination of artifacts like eyes movement and cardiac overlapping of cardiac position has been done. Tasks which was performed by the subjects include subtraction of two numbers without making any movement. Each trial has been commenced with the communication orally of 2-digit (subtrahend) and 4-digit (minuend) numbers like 42 and 3141, respectively. More details of the dataset can be found in [15]. As a ground truth labelling of dataset is done on the basis of performance report card which is available in the form of excel sheet with dataset. During data acquisition subjects were asked to perform arithmetic activity and nonstressed performer has performed 21 subtractions approximately and stressed performer has performed 7 subtractions in the given time. Number of nonstress performers in dataset is 26 and that of stress performers was 10. Dummy participants have been added to the dataset for nonstress category by replicating the data channelwise for an experimentation purpose with goal of balancing data for both categories. Age group of subjects is in range of 16–26; both male and female categories were included.

The total data of 36 subjects has been evaluated and has been given to the classifier by a robust and appropriate feature extraction approach. For labels in documentation for dataset [1], in the performance report of subjects with notation subject 0 to subject 35 which consist of name, age, gender, number of subtractions, and count quality **“G”** indicates good and **“B”** indicates bad, as mentioned in the excel file. Joining subject file with EEG data and name attribute created a labelled dataset file and those labels have been used as a ground truth for binary classification.

#### 2.1.1. Channel Selection

Channels included into study cover complete skull hemisphere ranging from frontal to occipital region: frontal position, 6 + 1 channels; temporal position, 4 channels; central position, 2 + 1 channels; parietal position, 2 + 1 channels; occipital position, 2 channels; behind the ear, 1 channel; and 1 ECG channel. Channel selection is done with objective in mind to investigate the affected areas so that precise marker can be identified in each category which definitely helps for identification of discrimination purpose of stress and nonstress biomarkers. Channel positions considered are illustrated in Figure 2.

### 2.2. Variational Mode Decomposition (VMD)

This decomposition method is robust for noise handling [35]. It is a process of decomposition of real valued input signal *f* into discrete number of subsignals also known as mode *u*_*k*_. Each mode is densely oriented towards its central frequency *w*_*k*_, which is determined during decomposition process. Each mode has a sparsity property which is being used while reconstructing the signal. Before decomposition sparsity of each mode has to be determined by bandwidth in spectral domain. To identify the bandwidth, three steps need to be followed which are given as follows:

(1) From each mode, Hilbert transform has been used to obtain the unilateral frequency domain.
(2) Subsequently, shift the frequency spectrum which has been obtained in step 1 to the baseband by integrating with an exponential tune to the respective centre frequency.
(3) Afterwards, apply *H*1 Gaussian smoothness to the demodulated signal for obtaining bandwidth given in
  (1) $$\begin{array}{c} \frac{\min}{\left\{u_{k}\right\},\left\{w_{k}\right\}}\left\{\sum_{k}\partial_{t}\left[\partial \left(t\right)+\frac{j}{\pi t}*u_{k}\left(t\right)\right]e^{-jw_{k}t}\right\}, \end{array}$$
where *u*_*k*_={*u*_1_,…, *u*_*k*_} and *w*_*k*_={*w*_1_,….*w*_*k*_}∑_*k*_*u*_*k*_=*f*.

The detailed behavior of variational mode decomposition (VMD) is as shown in Algorithm 1.

### 2.3. Poincare Plots (PPs)

PP of the modes obtained after VMD of EEG signals can provide favourable characteristic patterns for the classifications purpose. The PP of signal is defined as given in the equation below:

*x* (*t*) is a plotting of *X*(*t*) against *Y*(*t*) as shown in the following equations:

(2) $$\begin{array}{c} X\left(t\right)=x\left(t+1\right)-x\left(t\right), \end{array}$$

(3) $$\begin{array}{c} Y\left(t\right)=x\left(t+2\right)-x\left(t+1\right). \end{array}$$

This plot indicates the successive proportions against each other [36]. The resultant elliptical shape of plots portrayed from mode signifies the strong positive association between the consecutive data points, variability, and stochastic nature. As modes derived from signal are deviated towards central frequency, asymmetric area coverage is visible in PPs. Region coverage for the plot of the first eight modes is significantly higher than that of the other modes. Ten modes are obtained from the signal and evaluated but only first eight modes are considered for experimentation and the remaining two are excluded on the basis of significant area coverage as compared to the rest at central modes.

### 2.4. Features Extraction

Owing to the no stationary behavior of captured physiological signals, features obtained from the PPs are the area of the elliptic region, mean distance, and central tendency measure. PPs are designed from each mode obtained from variational mode decomposition, and for the calculation of area coverage of the elliptic shape of plots, the equations used are as follows:

(4) $$\begin{array}{c} S_{X}=\sqrt{\frac{1}{N}\sum_{i=0}^{N=1}X{\left(t\right)}^{2}}, \end{array}$$

(5) $$\begin{array}{c} S_{Y}=\sqrt{\frac{1}{N}\sum_{i=0}^{N=1}Y{\left(t\right)}^{2}}, \end{array}$$

(6) $$\begin{array}{c} S_{XY}=\frac{1}{N}\sum X\left(t\right)Y\left(t\right), \end{array}$$

(7) $$\begin{array}{c} {\text{Area}}_{\text{Ellipse}}=\pi ab, \end{array}$$

where $a=\text{major radius of poincare plots}\left(\sqrt{S_{X}^{2}+S_{Y}^{2}+D}\right.$), $b=\text{minor radius of poincare plots }\left(\sqrt{S_{X}^{2}+S_{Y}^{2}+D}\right.$), and $D=\sqrt{\left(S_{X}^{2}+S_{Y}^{2}\right)4\left(S_{X}^{2}S_{Y}^{2}+S_{XY}^{2}\right)}$.

Area computed from the PPs of EEG and ECG signals is used as a discriminative feature with 95% confidence. The details of area computation includes calculation of mean values *X*(*t*) and *Y*(*t*) as mentioned in equations (2) and (3).To compute plot parameter *D* compute mean values from equations (4)–(6). Ellipse area can be computed by equation (7). Mean and central tendency measure (CTM) of the PPs have been derived.

### 2.5. Classifier Used in Study

For the analysis of the robustness of the proposed approach, two classifiers have been tested which are multilayer perceptron neural network (MLPN) and support vector machine (SVM). First experimentation has been carried out with SVM. It is of category supervised learning and can be used for the purpose of data classification either at binary or at multiclass type. Each data point is indicated as *n*_*i*_ and requires *n*-dimensional space for plotting all data points in consideration. For classification purpose objective of an algorithm is to find an appropriate hyperplane where discrimination and segregation of correct data points are possible. In the condition where classification is not easily achievable kernelling is an option opted by SVM, which is a method to elevate lower dimensional input space to higher level. Unlike SVM MLPN has a capability of performing more complex operations and it had a tendency to approximate the input as it is integrated with nonlinear activation function.

As data is not separable linearly all the time MLPN does the error correction by using a backpropagation approach where initial set weights and biased get corrected in order to reduce the difference level between obtained and expected results. It is very useful for image classification approach as well. Authors have converted the data into labelled version by using the ground truth value as described in Section 2. Different numbers of layers have been experimented and suitable layers fixed are 10 neurons and 3 hidden layers at each level. Activation function employed is rectified linear unit (ReLU), various learning parameters are set to regularization, and alpha is decided to be at value 0.0001 as most studies have reported this value and it deems fit for our experimentation purpose as well. Number of iterations is set to 200. Adam optimizer is used for an optimization purpose and it has helped us to reach to the expected accuracy level for most of the subsets. In order to avoid very fast and very slow learning process we have selected the value 0.001 and kept it constant for experimentation. For SVM details the parameters selected are Cost *C*=0.90, Epsilon=0.1, RBF kernel=exp(−*g|x* − *y|*2), *g*=0.02, Iteration limit=100, and Numerical Tolerance=0.0010.

### 2.6. Performance Evaluation Measures

Performance evaluators mostly used are sensitivity, specificity, and accuracy which gives insight about training, validation, and testing phase in order to compute the variance and bias level of the classifier. In this work, performance of the proposed classifier has been evaluated by using three evaluation metrics such as accuracy, specificity, and sensitivity as represented in the following equations:

(8) $$\begin{array}{c} \text{sensitivity}\left(\text{SEN}\right)=\frac{\text{TP}}{\text{TP}+\text{FN}}*100, \end{array}$$

(9) $$\begin{array}{c} \text{specificity}\left(\text{SPE}\right)=\frac{\text{TN}}{\text{TN }+\text{ FP}}*100, \end{array}$$

(10) $$\begin{array}{c} \text{accuracy}\left(\text{ACC}\right)=\frac{\text{TTP }+\text{ TN}}{\text{TP }+\text{ TN }+\text{ FP }+\text{ FN}}*100, \end{array}$$

(11) $$\begin{array}{c} F1\text{ measure}=\frac{\text{TP}}{\text{TP}+\left(1/2\right)\left(\text{FP}+\text{FN}\right)}, \end{array}$$

(12) $$\begin{array}{c} \text{Kappa statistics}=\frac{\left(\text{percent agreement observed}\right)-\left(\text{percent agreement expected by chance alone}\right)}{100-\left(\text{percent expected by chance alone}\right)}, \end{array}$$

where *TN* and *TP* are the indicators to notify about how many data points have been correctly predicted by the classifier and *FP* and *FN* are the indicators to notify about how many data points have been incorrectly classified by the proposed classifier.

## 3. Results and Discussion

In this work, dataset used for the purpose of an experimentation and evaluation of stress classifier is available publicly [15]. These are recordings of EEG signals while performing the mental arithmetic task of finite duration.  Figure 3 shows the decomposition of signal by using VMD approach and its modes which are deviated towards the central frequency of the original input signal that proves the significance of an approach for better noise handling and its appropriateness for handling the lower frequency as compared to higher frequency components.

The PPs of first eight variational modes are shown in Figure 4. Plots for modes are clearly representing the varying area covered and it is more inclined towards lower frequency component mode as compared to higher frequency component mode. These are PPs of an EEG signal, for subject 1 (female, good performer) recorded for channel FP1, while performing mental arithmetic activity of 1 minute duration.

Features extracted described in Section 2, “Materials and Methods,” contributed for the designing of feature space. Extracted features from PPs contributed for the design of feature space and it is provided as an input to the SVM and multilayer perceptron neural network. Statistical significance of the extracted feature has been performed with Wilcoxon statistical significance test with *p* < 0.5. Extracted features are central tendency measure, mean distance, and area. The data generated for trail 1 and trail 2 for good performer female for channels FP1 and FP2 as listed in Table 1. Area coverage is the highest for middle modes as compared to initial and end position.

The Wilcoxon signed-rank test has been performed to verify the statistical significance of the features extracted with a confidence interval of 95 %.

To check robustness and more reliable performance evaluation of classifier data is provided to classifier in two ways for the first time, where 70%, 10%, 20% training, validation, and testing have been used by the split strategy to split the data and later k-fold data where value of *k* = 10 is selected. Only first eight modes have been used for the extraction of results. By considering all three features on 20% of test data from 36 subjects, the first to eight modes, binary classification results according to group selection of channels are listed in Table 2.  Table 3 summarizes results for the case of k-fold cross validation.

Modes extracted from EEG signals have displayed variable frequency behavior and because of tendency towards central frequency modes are fluctuating from lower to higher and vice versa. The central mode exhibited higher frequency components in comparison to initial and ending. Initial signal is decomposed into 10 modes but after 8th mode it has stopped exhibiting any variation in behavior and appears to be static in nature. Thus, only first 8 modes have been considered for an experimentation purpose. Remaining 8 nodes also exhibited some grouping characteristics; thus 3 groups with combination of 1–4 modes, 5–8 modes, and 1–8 modes are created and processed accordingly. As each subject consists of 21 channels decomposition has been done subjectwise and trialwise. For the decomposition of signals into modes it took approximately 2-3 mins and for designing PPs of mode it took approximately 3-4 mins for each subject. The range mentioned is because of different size of data points for trial 1 and trial 2 as explained in Section 2. For classification purpose two algorithms have been used, SVM and MLPN. The time taken for SVM is much more as compared to MLPN for binary classification of different subsets. By using k-fold, performance of classifier is improved compared to the intended percentage split base study. It is particularly notable for modes 1–4 and 1–8 but marginal for modes 5–8 except for the first set, good performer vs. bad performer. The better performance, in the case of k-fold cross validation, is attained because a higher percentage of data is used for the training purpose compared to the percentage split case. Authors main objective were to identify specific region of brain which exhibits significant behavior and can be used as marker for discrimination and thus subsets have been designed accordingly.

First subset is good vs. bad (combination of 20 EEG and 1 ECG channel) and subsequently 4 subsets are at regions frontal, temporal, central, and occipital. In addition to these five subsets 2 more subsets were tested for good vs. bad male and female but have not achieved any good classification accuracy as per gender and thus concluded that gender discrimination for performance is not possible through the designed approach and needs some other approach for the same as what also happened in case of subset for parietal region and has been excluded from an experimentation. Extracted modes exhibited the inconsistent and abrupt upsurge and/or fall, which can be taken care of by detection and removal of outliers before determining the PPs. Elliptic nature of plots varies/diminishes for different modes but only those modes have been considered for which plots have shown good elliptic curve and the rest were excluded for an experimentation purpose. Area covered by plots emerges as a combination of real imaginary numbers and we treated it in a form of absolute version. The reason for complex nature emerge is correct as plots of equations (4)–(6) involve root function and it is quite possible that the root results into negative number which emerges as a complex number.

Dataset consists of 21 channels but for an experimentation purpose initially only frontal channels were considered and subsequently temporal, central, and parietal ones were evaluated. At the end 20 EEG channels and 1 ECG channel were considered for experimentation. The feature map consists of channel, trail, mode, area, mean, and CTM of dimension 8 × 3 for each channel and subject. The first eight modes and their plots were generated for each of the undertaken channels. Later 3 features have been extracted from each consecutive plot. Wilcoxson signed-rank test has been performed to validate the statistical significance of the derived features with *p* < 0.5. The plot area has been considerably reduced at initial and end position of mode, which is a sign of less frequency contents of the underlying signal. In comparison, the mean derived from the PPs has shown even rise and steadiness that can be visible in case of central tendency measure.

The experimental results are noticeable for approximately all the subsets utilized for the classification. Most stress related studies reported for specific/limited channels [37–39]. The proposed approach for the stress classification has outperformed other existing methods [3, 40–43] by achieving 100% accuracy with minimum time of mental arithmetic activity and has also given an insight for the identification of marker lobewise (frontal, temporal, central, and occipital) rather than selection of channels in a generalized way. Our brain activity consists of interchange of ions between neurons which results into current flow through synaptic mode. Stress and emotions either generated naturally or in induced environment have a tendency to retain in the form of current flow. EEG device is meant to measure the voltage fluctuation that occurs because of the movement of the neuron and as it has tendency to retain some time; this is very effective way for the measure of positive and negative impact of any environmental situation on human brain [44–46]. Therefore, in this research work, an efficient and accurate classifier has been proposed with exceptional results for stress classification from EEG signals employing VMD, SVM, and multilayer perceptron. The maximum accuracy achieved at temporal and frontal lobe and in [47] was reported as category activation and discriminating area is observed at temporal lobe which is closely related with speech and nonspeech activity and as dataset [15] used study prototype which includes silent mental counting activity without any movement; the extracted results are relevant. Extracted results are more prominent at frontal and temporal region which is closely associated with concentration and focused mode of nature. The approach works nice for the intended dataset. In future the performance of the proposed method will be tested for other biomedical signals. The incorporation of event-driven methods can improve the performance of suggested solution in terms of computational effectiveness, compression, and power consumption [48–51]. Investigation of this approach is another prospect.

## 4. Conclusions

In this work, an attempt has been made to propose and explore the VMD approach and its Poincare plots for the classification of stress managing capability from the silent mental arithmetic activity. The VMD is a promising method for extracting the relevant features from the EEG + ECG signals. The resultant region of the Poincare plots has exhibited discriminating nature and varies widely for stress and nonstress category. Only the first six or seven modes provided the better classification accuracy for the comparative analysis of the stress. Signals accompanying with the activity have shown significant variability in comparison to the baseline activity for good performer while it has shown stability in case of bad performer and thus had a straightway more extensive influence on the Poincare plots. The area of good performer female has been significantly higher. The devised method has achieved the maximum accuracies of 100% for frontal and temporal lobes. The proposed scheme can be beneficial for the clinical identification of low- and high-dominance regions in the subjects. In future scope, the proposed method can be extended to study the classification of other brain conditions such as epilepsy, Alzheimer's, and depression. Because of the identified marker in frontal and temporal lobe this approach can be used as promising approach to implement in real time situation.

## Figures and Tables

**Figure 1:** The overall workflow of proposed method.

**Figure 2:** Channel positions considered in study: F =Frontal, C=Central, P=Parietal, O=Occipital, and T = Temporal.

**Figure 3:** VMD of the signal while performing mental arithmetic activity of 1 min duration for subject 1 (female, good performer), channel FP1.

**Figure 4:** PPs of the modes while performing mental arithmetic activity of 1 min duration for subject 1 (female, good performer), channel FP1.

**Algorithm 1:** Variational mode decomposition (VMD).

**Table 1:** Format of the feature map used in experimentation for channels FP1 and FP2 for trail 2.

Channel	Mode	Area	m (*r* = 0.5)	ctm (*r* = 0.5)	Target
*EEG Fp1*	1	2.53	0.93	0.19	1
*EEG Fp1*	2	37.39	0.20	0.26	1
*EEG Fp1*	3	63.25	0.13	0.29	1
*EEG Fp1*	4	11.44	0.31	0.25	1
*EEG Fp1*	5	4.78	0.41	0.24	1
*EEG Fp1*	6	48.82	0.16	0.28	1
*EEG Fp1*	7	12.03	0.28	0.28	1
*EEG Fp1*	8	33.35	0.22	0.26	1
*EEG Fp2*	1	3.19	0.85	0.21	1
*EEG Fp2*	2	4.70	0.56	0.24	1
*EEG Fp2*	3	22.77	0.26	0.25	1
*EEG Fp2*	4	27.51	0.28	0.24	1
*EEG Fp2*	5	27.43	0.23	0.25	1
*EEG Fp2*	6	22.22	0.24	0.26	1
*EEG Fp2*	7	29.60	0.21	0.28	1
*EEG Fp2*	8	1.77	0.42	0.27	1

**Table 2:** Classification results for the percentage split.

Sets	Statistical parameters	MPLN	SVM	MPLN	SVM	MPLN	SVM
		Modes 1-4		Modes 5-8		Modes 1-8	
Good performer vs. bad performer	Sensitivity	97.2	61.23	98	68.67	98	70.65
	Specificity	96.3	65.12	98	68.67	98	70.65
	Accuracy	97.2	61.23	98	68.67	98	70.65
	*F-*measure	0.95	0.65	0.97	0.57	1	0.69
	Kappa statistics	0.94	0.63	0.98	0.56	0.99	0.69

Good performer vs. bad performer (female)	Sensitivity	78.56	62.34	81.67	68.67	83.78	69.67
	Specificity	78.9	62.37	82.23	68.67	83.67	69.67
	Accuracy	76.56	62.78	81.78	68.67	83.67	69.67
	*F*-measure	0.67	0.64	0.82	0.65	0.87	0.67
	Kappa statistics	0.68	0.63	0.82	0.65	0.88	0.69

Good performer vs. bad performer (male)	Sensitivity	79.56	63.43	80.21	68.67	82.67	70.02
	Specificity	78.78	63.56	80.12	68.67	82.56	70.02
	Accuracy	78.67	63.56	80.32	68.67	82.67	70.02
	*F*-measure	0.87	0.65	0.79	0.68	0.83	0.69
	Kappa statistics	0.87	0.65	0.79	0.67	0.83	0.69

Good performer vs. bad performer (frontal region)	Sensitivity	98	70.78	98.45	70.67	99	72.67
	Specificity	98	78.78	98.45	70.67	99	72.67
	Accuracy	98	67.89	98.45	70.67	99	72.67
	F-measure	0.98	0.74	0.99	0.69	1	0.71
	Kappa statistics	1	0.78	1	0.7	1	0.71

Good performer vs. bad performer (temporal region)	Sensitivity	99.8	67.78	99.99	61.23	99.99	75.56
	Specificity	97.78	67.78	99.99	65.12	99.99	75.56
	Accuracy	99.8	67.78	99.99	61.23	99.99	75.56
	*F*-Measure	0.99	0.74	0.99	0.59	1	0.72
	Kappa statistics	1	0.74	1	0.59	1	0.76

Good performer vs. bad performer (occipital region)	Sensitivity	78.56	60	80.23	62.34	89.34	76.7
	Specificity	78.9	60	80.34	62.37	89.43	76.7
	Accuracy	76.56	60	80.32	62.78	89.34	76.7
	*F*-measure	0.88	0.58	0.89	0.62	0.85	0.74
	Kappa statistics	0.85	0.58	0.86	0.62	0.85	0.74

Good performer vs. bad performer (central region)	Sensitivity	75.78	64.67	79.78	63.43	80.56	68.78
	Specificity	76.89	64.67	79.56	63.56	80.56	68.78
	Accuracy	78.67	64	79.34	63.56	80.56	68.78
	*F*-measure	0.76	0.67	0.75	0.62	0.83	0.56
	Kappa statistics	0.78	0.65	0.78	0.62	0.83	0.56

**Table 3:** Classification results for the k-fold cross validation.

Sets	Statistical parameters	K-fold MPLN	K-fold SVM	K-fold MPLN	K-fold SVM	K-fold MPLN	K-fold SVM
		Modes 1-4		Modes 5-8		Modes 1-8	
Good performer vs. bad performer	Sensitivity	98.12	65.45	98.1	69	99.12	72.34
	Specificity	97	66	98	69	99	72.34
	Accuracy	97.56	63	98	69	99	72.34
	*F*-measure	0.98	0.7	0.97	0.59	1	0.7
	Kappa statistics	0.97	0.66	0.98	0.56	1	0.71

Good performer vs. bad performer (female)	Sensitivity	79.01	63.12	81.67	68.67	85.56	71.34
	Specificity	79.12	63.34	82.23	68.67	84	70
	Accuracy	77.45	63.45	81.78	68.67	84.02	71.78
	*F*-measure	0.69	0.68	0.82	0.65	0.89	0.68
	Kappa statistics	0.7	0.65	0.82	0.65	0.89	0.7

Good performer vs. bad performer (male)	Sensitivity	80.01	64.34	80.21	68.67	83	71
	Specificity	79.9	65.67	80.12	68.67	84	72
	Accuracy	79.12	64	80.32	68.67	84	71.34
	*F*-measure	0.89	0.65	0.79	0.68	0.86	0.72
	Kappa statistics	0.88	0.66	0.79	0.67	0.85	0.72

Good performer vs. bad performer (frontal region)	Sensitivity	98.23	71.01	98.45	70.67	100	75.23
	Specificity	98.45	79.23	98.45	70.67	100	73.23
	Accuracy	99.12	69	98.45	70.67	100	73.12
	*F*-Measure	0.99	0.76	0.99	0.69	1	0.72
	Kappa statistics	1	0.79	1	0.7	1	0.76

Good performer vs. bad performer (temporal region)	Sensitivity	99.82	68	99.99	61.23	100	76
	Specificity	98	68	99.99	65.12	100	78
	Accuracy	100	68	99.99	61.23	100	78
	*F*-measure	1	0.78	0.99	0.59	1	0.75
	Kappa statistics	1	0.76	1	0.59	1	0.78

Good performer vs. bad performer (occipital region)	Sensitivity	79.12	62.67	80.23	62.34	90	77
	Specificity	79	62	80.34	62.37	90	77
	Accuracy	77	61	80.32	62.78	90	77
	*F*-measure	0.9	0.6	0.89	0.62	0.87	0.78
	Kappa statistics	0.87	0.6	0.86	0.62	0.89	0.76

Good performer vs. bad performer (central region)	Sensitivity	76	65	79.78	63.43	82.12	69
	Specificity	77.78	65	79.56	63.56	82	69.12
	Accuracy	79.23	65	79.34	63.56	82	69
	*F*-measure	0.79	0.68	0.75	0.62	0.87	0.59
	Kappa statistics	0.79	0.66	0.78	0.62	0.86	0.59

## Data Availability

The dataset used in this paper is publicly available at https://physionet.org/content/eegmat/1.0.0/.
